This article has been retracted.

# Levels and Significance of Tumor Markers and Cytokines in Serum and Peritoneal Lavage Fluid of Patients with Peritoneal Metastasis of Gastric Cancer

**DOI:** 10.1155/2022/9528444

**Published:** 2022-06-02

**Authors:** Jianqi Yang, Wenmiao Cao, Enming Xing

**Affiliations:** Oncology Department of Northern Jiangsu People's Hospital Affiliated to Yangzhou University, 225000, China

## Abstract

The paper is written to investigate the levels and significance of tumor markers [carcinoembryonic antigen (CEA), carbohydrate antigen 125 (CA125), and carbohydrate antigen 19-9 (CA19-9)] and cytokines [interleukin-6 (IL-6), IL-4, and IL-2] in serum and peritoneal lavage fluid of patients with peritoneal metastasis of gastric cancer. For this research, 145 patients with gastric cancer treated in our hospital were divided into peritoneal metastasis group (*n* = 25), other metastasis group (*n* = 32), and nonmetastasis group (*n* = 88) according to the occurrence of metastasis. At the same time, the levels of serum tumor markers and cytokines and tumor markers and cytokines in intraoperative peritoneal lavage fluid were compared among the three groups. The results showed that the proportion of TNM stage III in peritoneal metastasis group and other metastasis group was 68.00% and 62.50%, respectively, and the proportion of tumor >5 cm was 64.00% and 59.38%, respectively, which was significantly higher than that in the control group. The 1-year survival rate of peritoneal metastasis group and other metastasis group was 44.00% and 40.63%, respectively, which was significantly lower than that of nonmetastasis group (*P* < 0.05).The serum levels of CEA, CA125, CA19-9, IL-6, IL-4, and IL-2 in peritoneal metastasis group and other metastasis group were higher than those in nonmetastasis group. The intraoperative peritoneal lavage fluid CEA, CA125, and IL-6 were 13.41 ± 3.72 ng/ml, 8.97 ± 1.33 U/ml, and 1.85 ± 0.44 pg/ml, respectively, which were higher than those in other metastasis groups and nonmetastasis groups (*P* < 0.05). There was no significant difference in the levels of CA19-9, IL-4, and IL-2 in peritoneal lavage fluid among peritoneal metastasis group, other metastasis groups, and nonmetastasis groups (*P* > 0.05); the areas under the ROC curve of intraoperative peritoneal lavage fluid CEA, CA125, and IL-6 in predicting peritoneal metastasis were 0.850, 0.902, and 0.806, respectively, *P* < 0.05. Thus, the conclusion is that peritoneal lavage fluid CEA, CA125, and IL-6 have certain application value in predicting and diagnosing peritoneal metastasis of gastric cancer, while the other indexes have no application value.

## 1. Introduction

Patients with advanced gastric cancer are prone to liver, peritoneal cavity and other important organ metastasis, and about 14%~43% of patients with gastric cancer have peritoneal metastasis [1]. Once peritoneal metastasis occurs, it will lead to malignant intestinal obstruction. The huge tumor load will lead to the rapid emergence of cachexia, systemic multiple organ failure, and the loss of the best time for antitumor treatment. The prognosis is so poor that the survival time is generally about 2~6 months [2]. Peritoneal dissemination is an inflammatory environment rich in inflammatory mediators, systemic chemotherapeutic drugs that cannot enter the abdominal cavity to cause peritoneal metastasis, and the effect of chemotherapy is not good. So far, the mechanism of peritoneal metastasis is not fully understood, so there is no exact treatment to alleviate the problem.

Relevant studies [3] suggest that the main factors affecting the prognosis of advanced gastric cancer are clinicopathological features, tumor markers, and cytokines. Tumor markers and cytokines can not only be used to screen high-risk groups, monitor recurrence and metastasis, as well as evaluate the efficacy of anti-tumor therapy but also predict the prognosis of a variety of malignant tumors. Peritoneal microenvironment is a hypoxic and high lactic acid environment. Some literatures suggest that intraperitoneal interleukin factor is considered as a predictor of poor survival and prognosis, which is helpful to judge whether patients have peritoneal metastasis and has guiding value in evaluating the condition and prognosis of patients [4]. Therefore, the significance of this study to investigate the levels of tumor markers and cytokines in serum, and peritoneal lavage fluid of patients with gastric cancer peritoneal metastasis is to explore the mechanism of peritoneal metastasis and to provide a basis for feasibility study. Peritoneal immunotherapy was followed up.

## 2. Research Objectives and Methods

### 2.1. General Information of Patients with Gastric Cancer

145 patients with gastric cancer treated in our hospital were included in the time range from January 2017 to January 2020. They met the following inclusion criteria: (1) confirmed by pathology; (2) radical gastrectomy in our hospital; (3) AJCC stage I~III; (4) no antitumor treatment before operation; and (5) informed consent of patients and their families. Meanwhile, they avoided the following exclusion criteria: (1) incomplete follow-up data; (2) tuberculosis, HIV, and other infections; and (3) accompanied by chronic obstructive pulmonary disease, coagulation dysfunction, and other serious diseases.

According to the occurrence of metastasis, the patients were divided into three groups: peritoneal metastasis group (*n* = 25), other metastasis group (*n* = 32), and nonmetastasis group (*n* = 88). There are 13 males and 12 females in peritoneal metastasis group, with an average age of 51.54 ± 8.22 years, ranging from 31 to 68 years; there are 20 males and 12 females in other metastasis groups, with an average age of 50.42 ± 9.15 years, ranging from 28 to 73 years old; there were 52 males and 36 females in the nonmetastasis group, with an average age of 51.22 ± 8.90 years, ranging from 30 to 74 years old. There was no significant difference in gender and age among the three groups (*P* > 0.05).

### 2.2. Inspection Index Method

Detection of serum indexes: took 3 ml of fasting venous blood of all patients within 24 h after admission, centrifuged at 3000 r/min for 10 min, and used the refrigerator at -80°C for testing after serum separation. The levels of serum CEA, CA125, CA19-9, IL-6, IL-4, and IL-2 were detected by enzyme-linked immunosorbent assay

Detection of peritoneal lavage fluid index: routine skin disinfection and local infiltration anesthesia after towel laying, needle core pulled out into abdominal cavity after anti-Michaelis point cannula puncture, and intraperitoneal infusion with 2000-3000 ml normal saline after connecting infusion. After proper activity, the patients were punctured to the abdominal cavity through the liver kidney space of the right upper abdomen under the guidance of ultrasound, and the abdominal lavage fluid was drained by cannula acupuncture to detect the levels of CEA, CA125, CA19-9, IL-6, IL-4, and IL-2

### 2.3. Statistical Processing

Spss22.0 software was used for analysis, and CEA, CA125, and other data are expressed by $\left(\bar{\chi }\pm \text{s}\right)$, and the differences between the groups are analyzed by *F* test. Gender and other data were expressed by frequency or percentage, and *χ*^2^ test was used to analyze the differences the between groups. ROC curve was used to analyze the predictive value. Inspection level *α* = 0.05.

## 3. Comparison Results of Various Research Data

### 3.1. Comparison of Clinical Data of Patients in each Group

The proportion of TNM stage III and the proportion of tumor size >5 cm in peritoneal metastasis group and other metastasis groups were significantly higher than those in nonmetastasis group (*P* < 0.05). There was no significant difference in sex, age, tumor location, and pathological type between peritoneal metastasis group, other metastasis group, and nonmetastasis group (*P* > 0.05). It is as shown in Table 1.

### 3.2. Comparison of 1-Year Survival Rate in each Group

The 1-year survival rate of peritoneal metastasis group and other metastasis group was 44.00% and 40.63%, respectively, which was significantly lower than that of nonmetastasis group (*P* < 0.05), as shown in Table 2.

### 3.3. Comparison of Preoperative Serum Tumor Markers and Cytokines in each Group

The levels of serum CEA, CA125, CA19-9, IL-6, IL-4, and IL-2 in peritoneal metastasis group and other metastasis groups were higher than those in nonmetastasis group (*P* < 0.05). There was no significant difference in serum levels of CEA, CA125, CA19-9, IL-6, IL-4, and IL-2 between peritoneal metastasis group and other metastasis groups (*P* > 0.05). It is as shown in Table 3.

### 3.4. Comparison of Tumor Markers and Cytokines in Intraoperative Peritoneal Lavage Fluid of Patients in each Group

The intraoperative peritoneal lavage fluid CEA, CA125, and IL-6 in peritoneal metastasis group were higher than those in other metastasis groups and nonmetastasis groups (*P* < 0.05); there was no significant difference in the intraoperative peritoneal lavage fluid CA19-9, IL-4, and IL-2 levels among peritoneal metastasis group, other metastasis groups, and nonmetastasis groups (*P* > 0.05). It is as shown in Table 4.

### 3.5. The Value of Intraoperative Peritoneal Lavage Fluid CEA, CA125, and IL-6 in Predicting Peritoneal Metastasis

The areas under the ROC curve of intraoperative peritoneal lavage fluid CEA, CA125, and IL-6 to predict peritoneal metastasis were 0.850, 0.902, and 0.806, respectively (*P* < 0.05), as shown in Figure 1, and the specific parameters are shown in Table 5.

## 4. Conclusion

Malignant tumor progression is the most common recurrence and metastasis, and peritoneal metastasis is one of the common biological behaviors in the recurrence and progression of gastric cancer. When it is diagnosed, it is mostly at the end of the disease [5, 6]. Gastric cancer patients with peritoneal metastasis lack typical symptoms in the early stage and are easy to be ignored. The results of this study show that there is no significant difference in gender, age, tumor location, and pathological type among peritoneal metastasis group, other metastasis groups, and nonmetastasis groups. This result is also consistent with previous clinical experience. In addition, this study also found that the proportion of TNM stage III and the proportion of tumor size >5 cm in peritoneal metastasis group and other metastasis groups were significantly higher than those in nonmetastasis group after comparison. Meanwhile, the one-year survival rates of peritoneal metastasis group and other metastasis groups were 44.00% and 40.63%, respectively, which were significantly lower than those in nonmetastasis group, suggesting that patients with advanced tumor were very prone to metastasis and the postoperative survival rate was significantly shortened. Therefore, in order to improve the prognosis of patients with peritoneal metastasis of gastric cancer, it is necessary to make early diagnosis and formulate and give targeted clinical intervention and systematic treatment.

CEA, CA125, and CA19-9 are important tumor markers. The changes of the above markers are commonly used in clinical work to detect the metastasis, recurrence, and curative effect evaluation of malignant tumors [7, 8]. IL-2, IL-4, and IL-6 are mainly separated from a variety of lymphocytes and nonlymphocytes. They are all multiactive cytokines, which can delay phagocytes from phagocytizing neutrophils and activate neutrophils, promote the activation, replication, and proliferation of B cells, and mediate the inflammatory response of the body [6, 9, 10]. The results showed that the levels of serum CEA, CA125, CA19-9, IL-6, IL-4, and IL-2 in peritoneal metastasis group and other metastasis groups were higher than those in nonmetastasis group, but there was no significant difference in serum indexes between peritoneal metastasis group and other metastasis groups. The above results suggest that the detection of serological tumor markers and cytokines is helpful to distinguish whether there is metastasis in patients with gastric cancer, but it is impossible to distinguish whether gastric cancer is peritoneal metastasis or other metastasis, and further examination and analysis are needed.

Traditional cytological examination of peritoneal lavage fluid is an important method for clinical detection of peritoneal free cancer cells. Relevant studies suggest that laparoscopic exploration and peritoneal lavage fluid cytology can find out whether there is peritoneal metastasis and the degree of peritoneal metastasis in gastric cancer patients with suspected peritoneal metastasis [11–13]. The results showed that CEA, CA125, and IL-6 in peritoneal lavage fluid in peritoneal metastasis group were higher than those in other metastasis groups and nonmetastasis groups, but there was no significant difference in other indexes. These results suggest that the tumor markers CEA and CA125 in peritoneal lavage fluid can indicate whether peritoneal metastasis occurs in patients with gastric cancer. Japanese scholars [14] found that even if there is no visible peritoneal metastasis in patients with gastric cancer, the possibility of micrometastasis cannot be ruled out. They advocated routine peritoneal lavage cytology and considered that peritoneal lavage cytology was positive and belonged to distant metastasis, which was consistent with the above results.

Further studies showed that the areas under the ROC curve of intraoperative peritoneal lavage fluid CEA, CA125, and IL-6 in predicting peritoneal metastasis were 0.850 and 0.902, respectively. It is suggested that peritoneal lavage fluid CEA, CA125, and IL-6 have certain application value in the prediction and diagnosis for peritoneal metastasis of gastric cancer. CEA is a carcinoembryonic antigen in embryo and fetus, which belongs to a protein complex rich in polysaccharides. Studies suggest that CEA is closely related to the prognosis of cancer. CA125 is a macromolecular carbohydrate protein complex, which does not rise significantly in mucinous epithelial carcinoma and granulosa cells but significantly increases in serous epithelial carcinoma and endometrioid carcinoma. It has become a commonly used tumor marker in clinic. Relevant literature [15] suggests that the peritoneal sensitivity of CA125 carcinoma to gastric cancer is more than 35%. However, some studies [16, 17] suggest that tumor markers may have a certain misdiagnosis rate and missed diagnosis rate in the diagnosis of gastric cancer metastasis, which may be due to the influence of comprehensive objective factors, such as individual physiological differences, and the characteristics of the tumor itself to the authenticity of the test results. Therefore, in clinical diagnosis, we also need to make a comprehensive judgment in combination with the actual clinical data, imaging, and other examination results of patients, so as to obtain more accurate diagnosis results, ensure that patients can receive symptomatic treatment, and improve the survival rate of patients.

In conclusion, CEA, CA125, and IL-6 in peritoneal lavage fluid have certain application value in the prediction and diagnosis of gastric cancer peritoneal metastasis, but other indexes have no application value.

## Figures and Tables

**Figure 1:** ROC curve analysis. ((a) Peritoneal lavage fluid CEA. (b) Peritoneal lavage fluid CA125. (c) Peritoneal lavage fluid IL-6).

**Table 1:** Comparison of clinical data of patients in each group.

Clinical data	Peritoneal metastasis group (*n* = 25)	Other metastasis group (*n* = 32)	Nonmetastasis group (*n* = 88)	F/c^2^	*P*
Gender					
Male	13 (52.00)	20 (62.50)	52 (59.09)	0.658	0.720
Female	12 (48.00)	12 (37.50)	36 (40.91)		
Years old	51.54 ± 8.22	50.42 ± 9.15	51.22 ± 8.90	1.032	0.687
TNM stage					
I~II	8 (32.00)	12 (37.50)	56 (63.64)	11.474	0.003
III	17 (68.00)	20 (62.50)	32 (36.36)		
Tumor site					
Upper 1/3	5 (20.00)	7 (21.88)	18 (20.45)	1.087	0.982
Middle 1/3	11 (44.00)	13 (40.63)	39 (44.32)		
Lower 1/3	7 (28.00)	11 (34.38)	25 (28.41)		
Cumulative two zones	2 (8.00)	1 (3.13)	6 (6.82)		
Tumor size					
≤5 cm	9 (36.00)	13 (40.63)	62 (70.45)	14.530	0.001
>5 cm	16 (64.00)	19 (59.38)	26 (29.55)		
Pathological type					
Adenocarcinoma	20 (80.00)	27 (84.38)	69 (78.41)	0.522	0.770
Other	5 (20.00)	5 (15.63)	19 (21.59)		

**Table 2:** Comparison of 1-year survival rate of each group.

Group	Number of cases	1-year survival rate (%)	*χ* ^2^	*P*
Peritoneal metastasis group	25	11 (44.00)	22.857	0
Other metastasis group	32	13 (40.63)		
Nonmetastasis group	88	71 (80.68)^ab^		

Meanwhile, ^a^compared with peritoneal metastasis group, *P* < 0.05; ^b^compared with other metastasis groups, *P* < 0.05.

**Table 3:** Comparison of preoperative serum tumor markers and cytokines in each group.

Group	Number of cases	CEA (ng/ml)	CA125 (U/ml)	CA19-9 (U/ml)	IL-6 (pg/ml)	IL-4 (ng/l)	IL-2 (ng/l)
Peritoneal metastasis group	25	140.45 ± 78.84	55.43 ± 21.03	140.41 ± 51.12	10.41 ± 2.01	12.24 ± 1.87	11.73 ± 1.95
Other metastasis group	32	138.82 ± 81.16	53.30 ± 18.87	137.73 ± 49.65	9.78 ± 1.84	11.70 ± 2.03	10.84 ± 2.00
Nonmetastasis group	88	11.54 ± 3.22^ab^	12.21 ± 2.46^ab^	21.15 ± 6.63^ab^	5.56 ± 1.16^ab^	6.10 ± 1.43^ab^	5.40 ± 1.21^ab^
*F*		34.541	31.106	27.844	14.541	12.265	11.037
*P*		0.000	0.000	0.000	0.000	0.000	0.000

Meanwhile, ^a^compared with peritoneal metastasis group, *P* < 0.05; ^b^compared with other metastasis groups, *P* < 0.05.

**Table 4:** Comparison of tumor markers and cytokines in intraoperative peritoneal lavage fluid of patients in each group.

Group	Number of cases	CEA (ng/ml)	CA125 (U/ml)	CA19-9 (U/ml)	IL-6 (pg/ml)	IL-4 (ng/l)	IL-2 (ng/l)
Peritoneal metastasis group	25	13.41 ± 3.72	8.97 ± 1.33	2.56 ± 0.89	1.85 ± 0.44	1.87 ± 0.27	1.15 ± 0.22
Other metastasis group	32	7.02 ± 1.44^a^	3.65 ± 1.03	2.40 ± 0.90	1.35 ± 0.30^a^	1.70 ± 0.32	1.13 ± 0.21
Nonmetastasis group	88	6.54 ± 1.22^a^	2.20 ± 1.10^ab^	2.37 ± 0.77	1.40 ± 0.31^a^	1.68 ± 0.29	1.12 ± 0.24
*F*		11.415	8.877	0.844	9.922	0.611	0.522
*P*		0.000	0.000	0.712	0.000	0.841	0.903

**Table 5:** Specific parameters of ROC curve.

Index	Area under curve	*P*	Truncation value	Sensitivity (%)	Specificity (%)
Peritoneal lavage fluid CEA	0.850	0.000	9.50 ng/ml	80.00	72.00
Peritoneal lavage fluid CA125	0.902	0.000	5.50 U/ml	85.00	78.50
Peritoneal lavage fluid IL-6	0.806	0.000	1.65 pg/ml	80.00	60.00

## Data Availability

The datasets used and analyzed during the current study are available from the corresponding author upon reasonable request.
